The article "Distribution of metals in coastal sediment from northwest sabah, Malaysia" was published in 2023. Journal: Heliyon.

# Distribution of metals in coastal sediment from northwest sabah, Malaysia

**DOI:** 10.1016/j.heliyon.2023.e13271

**Published:** 2023-01-27

**Authors:** Sin Yi Ling, Junaidi Asis, Baba Musta

**Affiliations:** a Faculty of Science and Natural Resources, Universiti Malaysia Sabah, 88400, Kota Kinabalu, Sabah, Malaysia; b Small Island Research Centre, Universiti Malaysia Sabah, 88400, Kota Kinabalu, Sabah, Malaysia

**Keywords:** Heavy metals, Major elements, Coastal sediment, Mineralogy, ICP-OES, Pearson correlation analysis

## Abstract

The type of minerals in sediments control the geochemical distribution of metals which serve as an indicator of the pollution status to the marine environment. The type of minerals was determined from X-ray diffraction (XRD) and scanning electron microscope (SEM) which shows the dominance of carbonate (calcite, aragonite, dolomite), silicate (quartz) and minor clay (illite, kaolinite) minerals. The elemental concentrations were also determined using the Inductively Coupled Plasma (ICP-OES) analysis that shows the major elements Ca > Fe > Mg > Al > Mn for all locations, whereas the heavy metals differ as Ni > Cr > Zn > Co > Pb, Cr > Ni > Zn > Pb > Co and Zn > Pb > Cr > Ni, respectively. The correlation between the major elements and heavy metals were also performed using the Pearson Correlation analysis via IBM SPSS which showed the positive Al–Fe–Mn correlation with the heavy metals but negative correlation with Ca. The correlations between the elements were influenced by the adsorption and precipitation of the major minerals in the sediment. The objective of this study is to determine the geochemical distribution of metals due to the influence of minerals in the coastal sediment of Kota Belud, Kudat and Mantanani Island. Therefore, this study could serve as a geochemical baseline data to understand the abundance of metals from the coastal region of northwest Sabah, Malaysia.

## 1 Introduction

Continental shelves, atolls or island arcs are the typical shallow water environments for massive carbonate formation near the coral reefs, while the pelagic deep-sea sediments above calcite compensation depth (CCD) zones also consist primarily of calcareous tests developed by marine biota in the water column [1]. Platforms for shallow-carbonates are mostly subjected at tropical to subtropical environment and accumulated at water depths shallower than 50 m, where high carbonate productivity are formed by benthic algae, mollusks and foraminifera [1,2]. In general, marine calcifying organisms show high calcification rates in response to the water column in alkalinity conditions which coprecipitate in the sediment matrices [3].

The article "Distribution of metals in coastal sediment from northwest sabah, Malaysia" was published in 2023. Journal: Heliyon.

Coastal sediments thus constitute the final medium of mineral deposits that can combine with heavy metals, via the adsorption/desorption kinetics, coprecipitation of solid phases, metal complexes or ionic binding and biological activity [[4], [5], [6], [7]]. The presence of heavy metals and their interactions with coastal sediment ultimately determines the accumulation and toxicity of metals that may lead to ocean pollution [8]. Generally, their toxicity and mobility are influenced by the total concentration and their mechanisms in the form of exchangeable fraction, carbonate fraction, Fe–Mn oxide (ferromanganese) fraction, organic fraction and residual fraction [9,10]. The carbonate minerals in coastal sediment hence play a major role to expediate or passivate the mechanisms, mobility, incorporation and distribution of metals to various parts of the sediments.

The major minerals in parent rocks or carbonate built-up platforms will also release metals or cause an elevated geochemical composition in sediment during natural weathering and erosional processes or from anthropogenic municipal wastes and industrial discharges [6,8,11]. The abundance and incorporation of heavy metals into coastal sediment is thus determined, whereby the gained data from present study is compared with existing quality guidelines to establish the range of metal concentrations of natural unpolluted coastal sediments. Therefore, this study acts as a baseline data to monitor the abundance of metals and pollution status of the shallow marine environment in the coastal region of northwest Sabah, Malaysia. The main objective of this study is to determine the geochemical distribution of metals due to the influence of minerals in the coastal sediment.

## 2 Materials and methods

### 2.1 Description of study area

This research was conducted in several coastal beaches that cover the northwest region of Sabah, particularly in Kudat, Kota Belud and Mantanani Island as shown in Fig. 1(a–c) and Fig. 2(a–c). The sampling locations are selected based on the contamination sources and different geological background from latitudes 6°18′N to 7°00′N and longitudes 116°15′E to 116°45′E. They are located in the intertidal region dominated by high sediment loadings from the shallow marine environment, river discharge, cascading events, marine biological production, and particle resuspension during storms or tidal waves from the South China Sea. High weathering of the source rocks due to tropical climate further increase the transport of weathered materials to the coastal regions.

**Fig. 1:** Base map for the study areas a) Kudat, b) Kota Belud and c) Mantanani Island from northwest of Sabah, Malaysia.a)Kudatb)Kota Beludc)Mantanani Island

**Fig. 2:** Geological map of a) Kudat, b) Kota Belud and c) Mantanani Island, from northwest of Sabah, Malaysia [23].

The article "Distribution of metals in coastal sediment from northwest sabah, Malaysia" was published in 2023. Journal: Heliyon.

The study areas consist of several rock formations, namely Ophiolite Basement, Chert-Spilite Formation, Crocker Formation, Kudat Formation, mélange or Wariu Formation, and Timohing Formation which contribute to the accumulation of Quaternary alluvial deposits in lowland areas or the ocean basins [[12], [13], [14], [15], [16], [17]]. The dismembered ophiolites and local geology also affect the metal abundance of present study and their spatial distribution. The recent carbonate build-ups from coral reefs and calcareous skeletal fragments from the marine environment that are washed ashore during the storm or tidal waves also contribute to the Quaternary alluvium and regulate the geochemical distribution of heavy metals in the coastal regions.

### 2.2 Sediment sampling

The equipment used in the sampling of sediment was washed using Merck Extran® MA2 soap and be first rinsed with tap water, then with deionized water. All glassware was soaked 24 h in 10% HNO_3_ acids and was rinsed with Milli Q® quality water. The sediment sampling was collected in transect along the coastal regions using a core sampler attached to a 1 m long PVC tube that was inserted vertically into the sediment surface. The tube was slowly removed and the bottom tube was sealed tightly with a Styrofoam stopper right when the tube was free from the bottom sediment. The core sampler was then removed from the tube and replaced by another Styrofoam stopper to tightly sealed the tube. A total of 27 vertical core samples were collected and taken to the laboratory to be horizontally extruded and subdivided into every 10 cm intervals that sum up to 153 sub-samplings. The sediment samples were then stored into airtight ziplock bags to avoid contamination and were kept at 4 °C inside a cooler box until further experimental analysis.

### 2.3 Experimental and statistical analysis

The air-dried sediment samples were ground and sieved through 63 μm mesh until 1 g fine-grained sediment fraction was collected. The aqua regia acid digestion method was conducted using the HCl:HNO_3_ mixture with 1:3 ratio based on the USEPA 6010D method and was then filtered through the Whatman 0.45 μm cellulose nitrate filter membrane to remove any suspended particles for cations analysis [18]. The Inductively-Coupled Plasma Spectrometry (ICP-OES) was performed using PerkinElmer Optima 5300 DV Spectrometer. This method was also reported by previous research to read the concentration readings of major elements Al, Ca, Fe, Mg and Mn, and heavy metals Co, Cr, Ni, Pb and Zn in the coastal sediment [19]. The readings were recorded by the spectrometer and raw data were processed and generated via the WinLab32 Software. The contamination level of heavy metals was then determined by comparing to the threshold values as stated in the sediment quality guidelines (SQGs) [20].

The article "Distribution of metals in coastal sediment from northwest sabah, Malaysia" was published in 2023. Journal: Heliyon.

XRD analysis was also performed to determine the major minerals in the sediment using Rigaku SmartLab2 device [21], whereas SEM analysis was also conducted to determine the mineral structures using the JEOL JSM-35 6100 microscope and Link AN 10/855 Analyser [22]. A 5 g of air-dried sediments were ground and sieved through 63 μm mesh for the XRD analysis, while another 5 g air-dried sediment was used for the SEM analysis. The IBM SPSS Statistics v28 software was then used to determine the correlation between the coefficients (Al, Ca, Fe, Mg, Mn, Co, Cr, Ni, Pb and Zn) using Pearson correlation analysis at significance levels of p < 0.01 and p < 0.05.

### 2.4 Quality assurance

A standard dilution stock solution of 100 mg/L was prepared to calibrate the instrument before carrying out ICP-OES analysis in compliance to the International Certified Reference Materials (CRM). All calculations for standard reference materials (SRM) analysis were done within a 80–120% accuracy to determine the suitability of the acid digestion method. All samples were performed in triplicate and were analyzed. Five reagent blanks were analyzed to determine the contamination and metal carry-over before proceed to the ICP-OES analysis.

## 3 Results and discussion

### 3.1 X-ray diffraction (XRD) analysis

This analysis is conducted for the mineralogical study of the sediment samples, whereby the diffractograms of the coastal sediments retrieved from 10 to 20 cm depth is shown in Fig. 3(a–c) from Kota Belud, Kudat and Mantanani Island, respectively. The primary mineralogy shows high carbonate content like aragonite, calcite and dolomite, followed by silicate minerals like quartz, and minor clay minerals like kaolinite and illite. From the diffractograms, the non-expandable illite and kaolinite are found only in the coastal sediments from Kota Belud and Kudat. The major minerals especially carbonates like calcite and aragonite might form small portions of amorphous calcium carbonate (ACC) phases in the sediments but were not detected in the X-Ray diffractometer.

**Fig. 3:** The spectra show minerals like aragonite (A), calcite (C), dolomite (D), illite (I), kaolinite (K) and quartz (Q) in the coastal sediments from a) Kota Belud, b) Kudat and c) Mantanani Island.

The type of minerals present controls the metal mobility, solubility, speciation, precipitation and sorption processes [24]. The abundant carbonate minerals are composed primarily of the coral community and calcareous shell remains from the marine environment [25]. The weathered materials from the fossiliferous limestone found in Kudat also contribute to the high carbonate content in the sediment. Limestone was known to release Mg, Ca and K metals into sediment [26]. The high MgO in soils might also have been leached from dolomite [CaMg(CO_3_)_2_] or magnesite [MgCO_3_] minerals [27].

The article "Distribution of metals in coastal sediment from northwest sabah, Malaysia" was published in 2023. Journal: Heliyon.

Precipitation and dissolution of crystalline carbonate phases such as calcite and aragonite may serve both as a sink and source to trap or remobilize metals such as Pb, Zn, Ni and Cr in natural environments [28,29]. Carbonate minerals have high sorption kinetics of metals which regulate their behavior, mobility and bioavailability in coastal sediment [30,31]. The heavy metals can substitute the carbonate phases that result in their depleted contents during their various interactions with the calcium carbonate in the sediment matrices [31]. Therefore, the higher bioavailability of Ca^2+^ facilitate the toxic metal removals by direct precipitation that form stable metal carbonates or by substitution with incorporating metals like Fe^2+^, Cu^2+^, Pb^2+^, Zn^2+^, Co^2+^, Ni^2+^ and Cr^2+^ in the calcium carbonate lattice structures [32,33].

Quartz is the primary mineral composition of onshore parent rocks that do not contribute to the natural source of heavy metals as it is resistant to weathering process and tend to exist in unactivated state [34,35]. However, the bicarbonate ions released during the weathering of carbonate minerals also increase the retention capacity of carbonate-buffer system which resist metal solubility and reduce their concentrations in the sediments [36,37]. This shows that carbonates increase the efficacy of metal assimilation from ingested particulate matter near the sediment-water interface and are thus often used for remediation and absorbent of metallic contaminants in soil or sediment [31,38,39]. Although the amorphous phases of CaCO_3_ were not detected in the XRD, they might still exist in small quantities and have the potential to combine with metals via adsorption and co-precipitation mechanisms [40].

The minor composition of clay minerals like kaolinite and illite exist in the silt/clay fractions of the sediment as part of the weathered parent materials from onshore rock outcrops. The clay minerals have layered aluminosilicates with large surface areas and active sites to bind with heavy metals Cr, Co, Ni, Pb and Zn, and facilitate their migration from the source to various parts of the sediments [24,41,42]. The adsorption mechanisms with metals include ion exchange, direct bonding and surface complexes between the clays with metal cations [43]. The decomposed organic ligands and humus in sediment also have high adsorption-desorption rate with metals to form stable organo-metal complexes, thereby increasing the metal extraction from the source and accumulate in lowlands or coastal shores [[44], [45], [46], [47]].

The article "Distribution of metals in coastal sediment from northwest sabah, Malaysia" was published in 2023. Journal: Heliyon.

### 3.2 Scanning electron microscope (SEM) analysis

Fig. 4(a–c) shows the SEM micrographs for the identification of major minerals, their morphology and structures in the coastal sediments retrieved from 10 to 20 cm depth as identified from Kota Belud, Kudat and Mantanani Island, respectively. The minerals identified are the carbonate minerals such as calcite or dolomite and aragonite, and clay minerals like illite and kaolinite. Fragments of marine skeletons were also found such as the foraminifera tests, corals and shells.

**Fig. 4:** The SEM micrographs show the minerals and skeletal fragments of marine organisms in coastal sediments of a) Kota Belud, b) Kudat and c) Mantanani Island.

Carbonate minerals are found as elongated aragonite columnar and rhombic calcite or dolomite in the coastal sediment. The nucleation of calcite in Kota Belud is seemingly more established in their rhombohedral morphology as some of the calcite surface in Kudat and Mantanani Island has been modified and became rather irregular, even though their general rhombohedral shapes were maintained. Amorphous calcium carbonates were also probably found more in Kudat and Mantanani Island sediments as compared to Kota Belud sediments. This could be due to the higher carbonate crystallite densities which retain their morphology and structure in the Kota Belud coastal region as shown in Fig. 3 [48]. This also suggests that the mineralization of calcium carbonates in Kudat and Mantanani Island have higher degree of structural flexibility to alter and conform into amorphous carbonate structures [49].

Relatively diverse structures of marine skeletal fragments from corals, shells and foraminifera tests are also found embedded near the amorphous calcium carbonates. The enriched carbonate minerals in the coastal sediment are thus contributed from the adjacent reef platforms composed of corals and skeletal remains of marine biogenic origins [16,50]. The high buffering capacity of carbonate minerals increase the adsorption mechanism with heavy metals to form stable and insoluble metal carbonates. This reduces the secondary pollution of heavy metals from remobilizing back into the marine environment [51].

Clusters of secondary clay minerals such as kaolinite and illite are also present. The kaolinite is detected in the form of stacked sheets and as loose intracrystalline structure while illite was detected in the form of both lamellar and flocculent structures. Clay content in the aluminosilicate precipitates is also formed by mineral recrystallization due to the alkalinity environment of the coastal shores [52]. The composition of clay minerals also affects the mobility and migration of heavy metals from the source to various parts of the coastal areas.

The article "Distribution of metals in coastal sediment from northwest sabah, Malaysia" was published in 2023. Journal: Heliyon.

### 3.3 Elemental *concentrations*

The concentrations of major elements and heavy metals were determined from the ICP-OES analysis. Table 1 shows the comparison of gained data from present study of Kota Belud, Kudat and Mantanani Island, with the range of natural unpolluted sediment guidelines established by the ANZECC/ARMCANZ legislations for coastal sediment. Kota Belud shows the overall highest elemental concentrations among the study areas, except Ca content. The total heavy metal contents are shown in Fig. 5, in which clearly denoting the influence of Ca concentration to the heavy metals. The distribution and abundance of the elemental concentrations were influenced by the major minerals present in the sediment as discussed in Section 3.1.

**Table 1:** Mean elemental concentration determined from ICP-OES analysis for each core samples from Northwest Sabah.

Study Area	Site	Core ID	Major Elements (mg/kg)						Heavy Metals (mg/kg)				
			Al	Ca	Fe	Mg	Mn		Co	Cr	Ni	Pb	Zn
Kota Belud	**1**	**K1A**	7000	4000	19,000	17,000	380		14	95	190	8.2	44
		**K1B**	8500	3900	21,000	20,000	540		17	98	230	7.6	43
	**2**	**K2A**	5800	2500	15,000	16,000	260		13	86	180	6.2	36
		**K2B**	6900	4700	19,000	20,000	380		16	110	210	8.1	40
		**K2A**	6200	3300	17,000	18,000	370		14	106	190	7.6	39
		**K2B**	6400	2800	18,000	18,000	320		15	94	200	7.4	41
	**3**	**K3A**	7400	3100	20,000	18,000	250		17	96	200	8.1	51
		**K3B**	9000	6200	21,000	15,000	320		18	79	170	9.6	51
	**4**	**K4A**	2600	350,000	4500	6300	140		1.8	9.0	12	2.5	19
		**K4B**	3400	230,000	5400	5600	100		1.6	8.2	9	4.3	22
**Min**			2600	2500	4500	5600	100		1.6	8.2	9.1	2.5	19
**Max**			9000	350,000	21,000	20,000	540		18	110	230	9.6	51
**Mean ± SD**			6300 ± 2000	62,000 ± 130,000	16,000 ± 6100	15,000 ± 5200	300 ± 130		12 ± 6.1	78 ± 38	150 ± 79	6.9 ± 2.1	38 ± 11
Kudat	**1**	**S1A**	1100	74,000	1800	4500	38		bdl	5.0	2.1	2.6	6.8
		**S1B**	1200	120,000	1900	6400	48		bdl	5.9	2.7	1.3	6.8
		**S1C**	870	76,000	1600	4200	31		bdl	5.6	2	2.9	6.3
		**S1D**	1300	110,000	1800	5200	40		bdl	14	7.2	1.9	6.6
		**S1E**	1600	160,000	2700	7700	54		0.08	11	5.7	1.5	9.3
		**S1F**	1500	110,000	2700	5600	47		0.16	13	8.2	2.1	7.1
	**2**	**S2A**	1700	190,000	1800	11,000	59		0.42	8.0	3.7	0.71	7.7
		**S2B**	1800	180,000	2300	9900	60		0.19	8.6	4.2	1.3	5.2
		**S2C**	2000	220,000	3000	11,000	68		0.29	8.1	3.9	0.4	5.9
		**S2D**	2100	260,000	3100	11,000	69		0.12	7.5	3.6	0.28	7.3
		**S2E**	2000	180,000	3100	9800	67		0.29	9.7	5.2	1.5	5.8
		**S2F**	2200	190,000	3000	9400	63		0.27	9.8	4.9	1.1	5.8
	**3**	**S3A**	950	310,000	1200	13,192	45		bdl	4.1	0.65	bdl	3.5
**Min**			870	74,000	1200	4200	31		0.08	4.1	0.65	0.28	3.5
**Max**			2200	310,000	3100	13,000	69		0.42	14	8.2	2.9	9.3
**Mean ± SD**			1600 ± 460	170,000 ± 70,000	2300 ± 660	8400 ± 2900	53 ± 12		0.23 ± 0.11	8.5 ± 3.0	4.2 ± 2.1	1.5 ± 0.80	6.5 ± 1.4
Mantanani Island	**1**	**M1A**	130	430,000	240	6100	18		bdl	5.0	0.29	2.1	39
		**M1B**	100	420,000	190	6700	17		bdl	5.9	0.13	2.6	8.0
	**2**	**M2A**	100	410,000	140	5600	13		bdl	5.6	1.3	9.0	9.3
		**M2B**	530	410,000	670	7700	26		bdl	14	6.0	25	15
**Min**			100	410,000	140	5600	13		–	5.0	0.13	2.1	8.0
**Max**			530	430,000	670	7700	26		–	14	6.0	25	39
**Mean ± SD**			200 ± 210	420,000 ± 13,000	300 ± 250	6500 ± 920	19 ± 5.8		–	5.8 ± 5.0	2.4 ± 2.8	8.3 ± 11	20 ± 14
**GUIDELINES**			**ANZECC/ARMCANZ** [20]		**ISQG-Low**				**-**	**80**	**21**	**50**	**200**
					**ISQG-High**				**-**	**370**	**52**	**220**	**410**

*bdl. Below detection limit.

The article "Distribution of metals in coastal sediment from northwest sabah, Malaysia" was published in 2023. Journal: Heliyon.

**Fig. 5:** Total heavy metals in the sediment core samples.

The concentration levels in Kota Belud show major elements Ca > Fe > Mg > Al > Mn, and heavy metals Ni > Cr > Zn > Co > Pb. The Ca concentration has the highest mean concentrations (62,000 mg/kg), followed by Fe (16,000 mg/kg), Mg (15,000 mg/kg), Al (6300 mg/kg), Mn (300 mg/kg), Ni (150 mg/kg), Cr (78 mg/kg), Zn (38 mg/kg), Co (12 mg/kg) and Pb (6.9 mg/kg). Although Ca has the highest mean value, the core samples from Station 1–3 has relatively lower Ca content than Station 4. As a result, the total heavy metal contents in Station 1 to 3 are relatively higher than Station 4 as shown in Fig. 5. The comparison with sediment guidelines shows that Ni and Cr contents have surpassed the trigger values as denoted by ISQG-low.

The concentration levels of Kudat show major elements Ca > Mg > Fe > Al > Mn, and heavy metals Cr > Ni > Zn > Pb > Co. The Ca concentration has the highest mean concentrations (170,000 mg/kg), followed by Mg (8400 mg/kg), Fe (2300 mg/kg), Al (1600 mg/kg), Mn (53 mg/kg), Cr (8.5 mg/kg), Ni (4.2 mg/kg), Zn (6.5 mg/kg), Pb (1.5 mg/kg) and Co (0.23 mg/kg). The current study demonstrates all heavy metals are within the permitted range of guidelines.

The concentration levels of Mantanani Island show major elements Ca > Mg > Fe > Al > Mn, and heavy metals Zn > Pb > Cr > Ni. The Ca concentration has the highest mean concentrations (420,000 mg/kg), followed by Mg (6, 500 mg/kg), Fe (300 mg/kg), Al (200 mg/kg), Mn (19 mg/kg), Zn (20 mg/kg), Pb (8.3 mg/kg), Cr (5.8 mg/kg) and Ni (2.4 mg/kg). The current study demonstrates all heavy metals are within the permitted range of guidelines.

The article "Distribution of metals in coastal sediment from northwest sabah, Malaysia" was published in 2023. Journal: Heliyon.

Toxic metals pollution in coastal sediment poses a major threat to the marine environment due to their toxicity, persistency, non-biodegradable and bio-accumulative nature that could disrupt the biological food chains of marine organisms [11,53]. Generally, their toxicity and mobility are influenced by the total concentration and their mechanisms in the form of exchangeable fraction, carbonate fraction, Fe–Mn oxide (ferromanganese) fraction, organic fraction and residual fraction [9,10]. According to the ANZECC/ARMCANZ [20] guidelines, all heavy metals from the gained data are within the allowable SQGs, except for Ni and Cr that has slightly exceed the SQGs in Kota Belud. The highly toxic nature of Ni and Cr can cause adverse impacts to the marine ecology and are also detrimental to human health if consumed [54].

The ultramafic parent rocks from Wariu formation or mélange of Kota Belud increase Ni and Cr concentration levels in the sediment [16,55]. Their abundance is also result from their high mobility and availability to be leached, transported and stored in the coastal banks or catchment region. The higher oxidation process in Kota Belud also increase the availability of Fe, Mn and Al elements that constitute a significant sink to form metal complexes with heavy metals Ni, Cr and Zn and increase their mobility to be transported from the parent soils to the coastal shores [56,57]. High sorbent phases of the Fe–Mn and Al–Mn oxides in the coatings within clay from Kota Belud also acts as a sponge-adsorbing system which further increase the adsorption kinetics with heavy metals and migrate to a further distance from the source [30]. Terrigenous materials such as land organisms, organic matter and other particulates also release heavy metals transported via channels, surface runoffs or leachate to the coastal environment [58].

However, the highly alkaline and saline properties along the coastal regions retain the heavy metals to accumulate in the sediment, thereby preventing the metals from remobilizing into the ocean water system as secondary pollution source [59]. The inclusion of shelled marine biota, benthic foraminifera, and coral deposits from the shallow marine ecology precipitate in-situ as calcium carbonate nodules or cement in the coastal sediments [16,31,60]. The high salinity and evaporation rates of seawater from marine environment also formed sedimentary dolomite [61,62]. Besides, the dolomites derived from limestone with high Ca and Mg base saturation levels also increase the carbonate mineral precipitation and alkalinity of sediment [63].

The article "Distribution of metals in coastal sediment from northwest sabah, Malaysia" was published in 2023. Journal: Heliyon.

The high Ca element in Kudat and Mantanani Island enriched by the autochthonous biogenic groups also form stable metal carbonates, which inhibit the metal mobility and reduce their ecotoxicity impact to the marine environment [[64], [65], [66]]. The correlation between Ca element and heavy metals were further interpreted using the Pearson correlation analysis to determine their association and potential sources in the study areas.

### 3.4 Pearson *Correlation* analysis

The correlation between the major elements and heavy metals could interpret their potential sources and association to form metal compounds for the distribution and migration of heavy metals from the source to the coastal shores in lowland areas [67,68]. Table 2 shows the association between the major elements and heavy metals at significance level of p < 0.01 and p < 0.05. The coastal sediment of Kota Belud shows a strong positive Fe–Al correlation (0.7 ≤ r < 1) but strong negative Ca correlation (−0.7 ≤ r < −1) with heavy metals like Co, Cr, Ni, Pb and Zn. Other major elements like Mg and Mn are also strongly positive correlated to heavy metals. Besides, the individual heavy metals also show strong positive correlation to one another.

**Table 2:** Pearson correlation analysis for the elements in the study areas.

Kota Belud										
Element	Al	Ca	Fe	Mg	Mn	Co	Cr	Ni	Pb	Zn
**Al**	1									
**Ca**	−0.864**	1								
**Fe**	0.962**	−0.940**	1							
**Mg**	0.805**	−0.915**	0.919**	1						
**Mn**	0.786**	−0.731^a^	0.818**	0.839**	1					
**Co**	0.950**	−0.937**	0.988**	0.922**	0.775**	1				
**Cr**	0.799**	−0.941**	0.922**	0.986**	0.800**	0.922**	1			
**Ni**	0.863**	−0.953**	0.958**	0.987**	0.834**	0.960**	0.980**	1		
**Pb**	0.943**	−0.913**	0.951**	0.813**	0.695^a^	0.934**	0.847**	0.857**	1	
**Zn**	0.948**	−0.876**	0.955**	0.800**	0.636^a^	0.955**	0.815**	0.860**	0.950**	1
**Kudat**										
**Element**	**Al**	**Ca**	**Fe**	**Mg**	**Mn**	**Co**	**Cr**	**Ni**	**Pb**	**Zn**
**Al**	1									
**Ca**	0.424	1								
**Fe**	0.868**	0.195	1							
**Mg**	0.517	0.968**	0.224	1						
**Mn**	0.935**	0.626^a^	0.782**	0.720**	1					
**Co**	0.260	0.127	−0.397	0.455	0.283	1				
**Cr**	0.366	−0.225	0.448	−0.227	0.163	−0.367	1			
**Ni**	0.381	−0.276	0.518	−0.273	0.181	−0.389	0.980**	1		
**Pb**	−0.796**	−0.921**	−0.557	−0.904**	−0.877**	−0.287	−0.010	0.013	1	
**Zn**	0.134	−0.431	0.256	−0.405	0.021	−0.361	0.377	0.425	−0.018	1
**Mantanani Island**										
**Element**	**Al**	**Ca**	**Fe**	**Mg**	**Mn**	**Co**	**Cr**	**Ni**	**Pb**	**Zn**
**Al**	1									
**Ca**	−0.440^a^	1								
**Fe**	0.985**	−0.444^a^	1							
**Mg**	0.171	−0.068	0.150	1						
**Mn**	0.666**	−0.204	0.668**	0.623**	1					
**Co**	–	–	–	–	–	–				
**Cr**	0.990**	−0.498^a^	0.973**	0.143	0.610**	–	1			
**Ni**	0.989**	−0.565^a^	0.977**	0.005	0.570^a^	–	0.999**	1		
**Pb**	0.916**	−0.437^a^	0.867**	0.108	0.477^a^	–	0.931**	0.918**	1	
**Zn**	−0.061	0.174	−0.008	−0.742**	−0.146	–	−0.080	0.014	−0.104	1

a Significance at p < 0.05 **significance at p < 0.01.

The article "Distribution of metals in coastal sediment from northwest sabah, Malaysia" was published in 2023. Journal: Heliyon.

Coastal sediment of Kudat shows strong positive correlation of Al with Fe and Mn, but strong negative correlation with Pb. Both Ca and Fe are positively correlated to Mg, while Fe and Mg are positively correlated to Mn. Among the heavy metals, only Cr is strongly positive correlated to Ni, but Pb is strongly negative correlated to the major elements Al, Ca, Mg and Mn. The others do not show any significant correlation.

Coastal sediment of Mantanani Island shows a strong positive correlation of Al with Fe, Cr, Ni and Pb, whereas Ca shows a moderate negative correlation (−0.4 ≤ r < −0.7) with Al, Fe, Ni and Pb. Fe also shows a strong positive correlation with Cr, Ni and Pb metals, but Mg shows a strong negative correlation with Zn. Mn shows moderate positive correlation with Al, Fe, Mg, Cr, Ni and Pb. Other heavy metals Cr, Ni and Pb are strongly positive correlated to one another.

The strong positive Al–Fe–Mn association suggest they are released from the weathering of similar source rocks during the redox process, such as the sedimentary rocks or dismembered ophiolite complex [16,69]. The strong Pb–Zn correlation further suggest they originate from sandstone, shale and calcareous siltstone of the Crocker and Kudat Formations, or cherts of the Chert-Spilite Formation [70,71]. Heavy metals correlate directly with the Al, Fe and Mn elements which indicate the constitution of primary carriers to transport the metals from the source through direct ionic bonding, metal cation exchange, redox potential or forming metal compounds in the sediment [30,72].

The strong positive Co–Cr–Ni association from Kota Belud also suggest they originate from the pedogenesis of serpentinized ultrabasic rocks from the Wariu Formation or dismembered ophiolitic rocks [55,73,74]. The relatively higher adsorptive kinetics and exchange capability of Cr, Ni and Zn metals as compared to Co and Pb metals, also facilitate their distribution and increase their abundance in the coasts [75]. Other heavy metals having no association are also enriched by human activities in the industry, agriculture, domestic or other socio-economic sectors that may deteriorate the sediment quality [11,76]. Heavy metals are also released from the natural emission of hydrothermal activities from the marine environment that influence their abundance and distribution along the coastal shores [77,78].

The article "Distribution of metals in coastal sediment from northwest sabah, Malaysia" was published in 2023. Journal: Heliyon.

Studies found that most metals are positively correlated to Fe in marine sediment due to the association with detrital particles but weak or negatively correlated with Ca as the calcareous shells act as diluents for most of the metals [[79], [80], [81]]. The weak correlations with Ca further indicate that carbonates are less significant binding phase for heavy metals as compared to Fe and other mineral elements in the sediment matrices [82,83]. Therefore, the negative correlation of metals with calcium concentrations depict the reduction of heavy metals due to carbonate precipitation to form stable metal carbonate which trap and inhibit their leachability, mobility and distribution [64,66,84]. The predominance of quartz with high crystallinity in the sand fraction also might cause difficulty when interpreting the possible mineral sources of heavy metals in sediments, that result in the weak or no correlations [85].

The high buffering capacity and adsorptive kinetics of Ca also constitute the primary sink or storage for heavy metals from remobilizing and leaching into the seawater as secondary pollutants [51,86]. Therefore, heavy metals are effectively retained and precipitate to the carbonate surfaces at low metal concentrations by the chemisorption mechanisms, which originate from the shallow marine corals or shelled marine biota [16,30]. The strong positive Ca–Mg association from Kudat also indicated they originate from dolomite or limestone of the Kudat Formation [87].

## 4 Conclusion

In conclusion, the overall mean of elemental concentrations from the three study regions showed the decreasing range of Ca (62,000–420,000 mg/kg) > Fe (300–16,000 mg/kg) > Mg (6500–15,000 mg/kg) > Al (200–6300 mg/kg) > Mn (19–300 mg/kg) > Ni (2.4–150 mg/kg) > Cr (5.8–78 mg/kg) > Zn (6.5–38 mg/kg) > Co (0.23–12 mg/kg) > Pb (1.5–6.9 mg/kg). The gained data were compared to the guidelines established by ANZECC/ARMCANZ, which showed Ni and Cr have surpassed the normal range for coastal sediment in Kota Belud. The present study also showed the domination of carbonate (calcite, aragonite, dolomite), silicate (quartz) and minor clay (illite, kaolinite) minerals that influence the migration, accumulation and distribution of metals in the coastal sediment. The distribution of metals due to the influence of carbonate minerals is also determined from strong positive Al–Fe–Mn correlation but the strong negative Ca correlation with the heavy metals. Therefore, this study serves as a geochemical baseline data to monitor the current status and distribution of metals from the coastal region of northwest Sabah, Malaysia.

The article "Distribution of metals in coastal sediment from northwest sabah, Malaysia" was published in 2023. Journal: Heliyon.

## Declarations

### Credit author statement

Baba Musta: Conceived and designed the experiments; Analyzed and interpreted the data; Contributed reagents, materials, analysis tools or data; Wrote the paper.Ling Sin Yi: Performed the experiments; Analyzed and interpreted the data; Wrote the paper.Junaidi Asis: Contributed reagents, materials, analysis tools or data.

### Funding statement

Prof Dr Baba Musta was supported by 10.13039/501100003093Ministry of Higher Education, Malaysia [TR@M001-2019].

### Data availability statement

No data was used for the research described in the article.

## Declaration of competing interest

The authors declare that they have no known competing financial interests or personal relationships that could have appeared to influence the work reported in this paper.
